# Astragaloside IV inhibits platelet-derived growth factor-BB-stimulated proliferation and migration of vascular smooth muscle cells via the inhibition of p38 MAPK signaling

**DOI:** 10.3892/etm.2014.1905

**Published:** 2014-08-14

**Authors:** ZHUO CHEN, YING CAI, WENLIANG ZHANG, XINZHOU LIU, SUIXIN LIU

**Affiliations:** Cardiac Rehabilitation Center, Department of Rehabilitation, Xiangya Hospital of Central South University, Changsha, Hunan 410008, P.R. China

**Keywords:** astragaloside IV, platelet-derived growth factor, vascular smooth muscle cell, proliferation, migration

## Abstract

Astragaloside IV (AS-IV), the major active component extracted from *Astragalus membranaceus*, has been demonstrated to exhibit protective effects on the cardiovascular, immune, digestive and nervous systems; thus, has been widely used in traditional Chinese medicine. Abnormal proliferation and migration of vascular smooth muscle cells (VSMCs) is closely associated with the initiation and progression of cardiovascular diseases, including atherosclerosis and restenosis. However, the effects of AS-IV on VSMCs remain unknown. For the first time, the present study demonstrated that AS-IV markedly suppressed platelet-derived growth factor (PDGF)-BB-stimulated cellular proliferation and migration of HDMEC-a human dermal VSMCs (HDVSMCs). Further investigation into the underlying molecular mechanisms demonstrated that the administration of AS-IV attenuated the PDGF-BB-stimulated switch of HDVSMCs into a proliferative phenotype. Furthermore, AS-IV inhibited the PDGF-BB-induced expression of cell cycle-associated proteins, as well as the upregulation of matrix metalloproteinase (MMP)2, but not MMP9. In addition, AS-IV was shown to downregulate the activation of p38 mitogen-activated protein kinase (MAPK) signaling induced by PDGF-BB in HDVSMCs. Therefore, the observations of the present study indicate that AS-IV inhibits PDGF-BB-stimulated VSMC proliferation and migration, possibly by inhibiting the activation of the p38 MAPK signaling pathway. Thus, AS-IV may be useful for the treatment of vascular diseases.

## Introduction

Radix Astragali Mongolici is the dried root of the leguminous plant, Mongolia Astragalus, which has been used in traditional Chinese medicine for the treatment of hepatitis, kidney disease, cardiovascular disorders and skin diseases for more than two thousand years (1). Astragaloside IV (AS-IV) is the main compound extracted from the astragalus root, and has been recently demonstrated to exhibit various pharmacological effects on the liver, nervous system, hematopoietic system, endocrine system, cardiac function, metabolism of collagen and organ immune system (1). Furthermore, AS-IV has been shown to promote the proliferation of human umbilical vein endothelial cells, as well as the formation of tube-like structures *in vitro* (2). In addition, AS-IV has been reported to stimulate angiogenesis via the phosphoinositide 3-kinase/Akt, janus kinase 2/signal transducer and activator of transcription 3 and extracellular-signal-regulated kinase 1/2 pathways (3,4). These observations indicate that AS-IV may have important effects on cardiovascular disorders.

Cardiovascular disorders often involve the abnormal proliferation and migration of vascular smooth muscle cells (VSMCs) in arterial walls, which has been reported to play crucial roles in the initiation and progression of arteriosclerosis and restenosis following percutaneous coronary intervention (PCI) (5–7). VSMCs remain in a quiescent state under physiological conditions; however, the cells undergo phenotypic changes to an uncontrolled proliferative and migratory state in response to various stimuli, including vascular damage and inflammation (8,9). Following vascular injury, such as angioplasty, numerous inflammatory cytokines are released by endothelial cells and macrophages, which further stimulate the phenotype switch of VSMCs to a proliferative and migratory state (10).

Furthermore, platelet-derived growth factor (PDGF) and its receptors are major mitogens for VSMCs (11). In response to vascular injury, the production of PDGF-BB is significantly upregulated, which further stimulates the proliferation and migration of VSMCs (12). In addition, PDGF-BB has been widely used for stimulating the VSMC phenotype switch (13,14). However, the detailed effects of AS-IV on PDGF-BB-stimulated VSMCs remain unclear.

As an antiproliferative and antimigratory agent for VSMCs, AS-IV demonstrates promise for the treatment of cardiovascular disorders. Thus, the aim of the present study was to investigate the effects of AS-IV on VSMC proliferation and migration, as well as the underlying mechanisms. Our findings for the first time reported the suppressive effects of AS-IV on PDGF-BB-induced cellular proliferation and migration in HDMEC-a human dermal VSMCs (HDVSMCs). We also found that the molecular mechanism by which AS-IV inhibited PDGF-BB-stimulated HDVSMC proliferation and migration was closely associated with the downregulation of p38 MAPK signaling pathway.

## Materials and methods

### Materials and agents

Dulbecco’s modified Eagle’s medium (DMEM)/F12 medium and fetal bovine serum (FBS) were purchased from Invitrogen Life Technologies (Carlsbad, CA, USA). Recombinant human PDGF-BB was purchased from ACROBiosystems, Inc. (Newark, DE, USA) and AS-IV was purchased from Tauto Biotech (Shanghai, China). Dimethyl sulfoxide (DMSO) and MTT were purchased from Sigma-Aldrich (St. Louis, MO, USA). Mouse anti-smoothelin, anti-α-smooth muscle actin (α-SMA), anti-desmin, anti-phospho-p38 mitogen-activated protein kinase (MAPK), anti-p38 MAPK, anti-matrix metalloproteinase (MMP)2, anti-MMP9 and anti-GAPDH antibodies, as well as a goat anti-mouse secondary antibody, were obtained from Abcam (Cambridge, UK).

### Cell culture

An HDMEC-a HDVSMC line was purchased from ScienCell Research Laboratories (Carlsbad, CA, USA) and cultured in DMEM/F12 medium supplemented with 10% FBS at 37°C in a humidified atmosphere of 95% air and 5% CO_2_.

### Cell proliferation assay

Prior to the cell proliferation assay, HDVSMCs were cultured to 60% confluence in 96-well plates, and then serum-starved for 24 h. In the PDGF-BB group, HDVSMCs were treated with 30 ng/ml PDGF-BB for 6, 12, 24 and 48 h. In the PDGF-BB + AS-IV group, HDVSMCs were treated with 30 ng/ml PDGF-BB and 10 μM AS-IV for 6, 12, 24 and 48 h. HDVSMCs without any treatment were used as a control.

To analyze the cell proliferation rate in each group, MTT assays were performed. In each well, 0.5 μg/ml MTT was added to the medium and then incubated for 3 h. Next, the medium was removed and 100 μl DMSO was added. The 96-well plate was gently rotated for 15 min to dissolve the precipitation. Absorbance values were measured at 570 nm using a microplate reader (Bio-Rad, Hercules, CA, USA), from which the proliferation rate in each group was determined.

### HDVSMC migration assay

Cell migration rates in each group were examined using a Costar 24-well chamber (Corning, NY, USA). In brief, cell suspensions (5×10^5^ cells/ml) were prepared in DMEM/F12 medium. In accordance with the manufacturer’s instructions, 500 μl DMEM/F12 with 10% FBS was added to the lower chamber, and 300 μl cell suspension was added to the upper chamber. In the PDGF-BB group, 30 ng/ml PDGF-BB was added to the lower wells, while in the PDGF-BB + AS-IV group, 30 ng/ml PDGF-BB and 10 μM AS-IV were added to the lower wells. After 24 h incubation at 37°C with 5% CO_2_, the cells that had not passed through the membrane were removed, while the cells that had transferred across the membrane were stained with crystal violet dye for 30 min. These cells were then rinsed with water and dried in air. The stained cells in five randomly selected fields were counted.

### Western blot analysis

Western blot analysis was used to determine protein expression levels. Briefly, cells were lysed in pre-cooled radioimmunoprecipitation assay buffer and the protein concentration was examined using a bicinchoninic acid protein assay kit (Thermo Fisher Scientific, Waltham, MA, USA). For the determination of protein expression, the protein was separated by 10% SDS-PAGE and transferred to a polyvinylidene fluoride membrane. Next, the membrane was blocked in 5% nonfat milk in phosphate-buffered saline at 4°C overnight, followed by incubation with the specific primary antibodies for 3 h at room temperature. The membrane was then incubated with the goat anti-mouse secondary antibody. Immune complexes were detected using an enhanced chemiluminescence kit (Thermo Fisher Scientific).

### Statistical analysis

All the data are expressed as the mean ± standard deviation of three independent experiments. One-way analysis of variance followed by Fisher’s least significant difference post-hoc test were used to perform statistical analysis using SPSS 19.0 software (SPSS, Inc., Chicago, IL, USA). P<0.05 was considered to indicate a statistically significant difference.

## Results

### AS-IV inhibits PDGF-BB-stimulated VSMC proliferation

The effect of AS-IV on PDGF-BB-induced VSMC proliferation was analyzed by performing MTT assays. The results demonstrated that PDGF-BB treatment significantly promoted the cellular proliferation of HDVSMCs; however, pretreatment with AS-IV markedly attenuated the effect of PDGF-BB on VSMC proliferation (Fig. 1). These observations indicated that AS-IV exhibited a suppressive effect on PDGF-BB-stimulated VSMC proliferation.

### AS-IV inhibits PDGF-BB-induced expression of cell cycle-associated proteins in HDVSMCs

As AS-IV exhibited a suppressive effect on PDGF-BB stimulated VSMC proliferation, it was hypothesized that the role of AS-IV in HDVSMCs may be associated with the expression of cell cycle-associated proteins. Therefore, the protein expression levels of cyclin-dependent kinase (CDK)2, CDK4, cyclin D1 and cyclin E were analyzed using western blot analysis. The results revealed that the administration of PDGF-BB markedly upregulated the protein expression levels of these cell cycle-associated proteins in the HDVSMCs, and this was significantly attenuated by pretreatment with AS-IV (Fig. 2). These observations indicated that AS-IV suppressed PDGF-BB-induced upregulation of cell cycle-associated proteins in HDVSMCs.

### AS-IV inhibits the PDGF-BB-induced phenotype switch of HDVSMCs

Under physiological conditions, HDVSMCs are known to have a differentiated phenotype, while under specific stimulations, including vascular damage or inflammatory responses, HDVSMCs can switch into a proliferative phenotype. Accordingly, the expression levels of three markers for the differentiated phenotype of HDVSMCs, smoothelin, α-SMA and desmin, were analyzed. The results showed that administration of PDGF-BB significantly downregulated the protein expression levels of these three markers in the HDVSMCs, indicating that the HDVSMCs had dedifferentiated into a proliferative phenotype (Fig. 3). However, pretreatment with AS-IV markedly attenuated the downregulation of α-SMA, smoothelin and desmin expression levels induced by PDGF-BB (Fig. 3). These observations indicated that AS-IV exhibited an inhibitory effect on the PDGF-BB-induced phenotype switch in HDVSMC.

### AS-IV inhibits PDGF-BB-stimulated VSMC migration

The effect of AS-IV on PDGF-BB-stimulated HDVSMC migration was investigated using a Transwell assay. The results demonstrated that administration of PDGF-BB markedly promoted VSMC migration when compared with the control HDVSMCs that did not receive any treatment (Fig. 4). However, pretreatment with AS-IV significantly attenuated the effect of PDGF-BB on VSMC migration (Fig. 4). The observations indicated that AS-IV plays a suppressive role in PDGF-BB-stimulated VSMC migration.

### AS-IV inhibits the PDGF-BB-induced upregulation of MMP2 in HDVSMCs

As MMP2 and MMP9 are key factors in the regulation of cellular migration, the expression levels of these two proteins were analyzed in each group. As shown in Fig. 5, the protein expression levels of MMP2 and MMP9 were significantly increased following PDGF-BB treatment. However, pretreatment with AS-IV reversed the upregulation of MMP2, but showed no effect on MMP9 (Fig. 5). These observations indicated that a potential method underlying the AS-IV inhibition of PDGF-BB-induced VSMC migration may be the suppression of MMP2 protein expression.

### AS-IV suppresses PDGF-BB-induced activation of p38 MAPK signaling in HDVSMCs

Since the expression levels of cell cycle-associated proteins and MMPs are directly mediated by p38 MAPK signaling, and this signaling pathway also plays a key role in the regulation of VSMC proliferation and migration under stimulation, including vascular damage and inflammation (15), the activity of p38 MAPK signaling in HDVSMCs was further investigated using western blot analysis. As demonstrated in Fig. 6, the expression of phospho-p38 MAPK in PDGF-BB-stimulated HDVSMCs was markedly increased compared with the HDVSMCs in the control group; however, pretreatment with AS-IV effectively suppressed the activation of p38 MAPK signaling stimulated by PDGF-BB. These observations indicated that AS-IV inhibited PDGF-BB-induced VSMC proliferation and migration via inhibiting the activation of p38 MAPK signaling.

## Discussion

VSMCs are the stromal cells of the vascular wall. They play a crucial role in the physiological and pathological processes of the vascular wall due to the continual exposure to the biochemical components in the blood compartment. Abnormal proliferation and migration of VSMCs in arterial walls is important for the initiation and progression of arteriosclerosis and restenosis. In the present study, AS-IV was found to exhibit a suppressive effect on PDGF-BB-stimulated HDVSMC proliferation and migration by inhibiting the switch of HDVSMCs into a proliferative phenotype, the expression of cell cycle-associated proteins and the upregulation of MMP2. In addition, AS-IV was shown to suppress the activation of p38 MAPK signaling induced by PDGF-BB in HDVSMCs. For the first time, the observations reveal the potential molecular mechanisms underlying the protective effects of AS-IV on VSMCs.

Vascular injury stimulates the production and secretion of inflammatory factors and cytokines, and these factors further promote VSMC proliferation and migration, which play important roles in the initiation of neointima formation (7). In addition, neointima formation is an important pathological event in atherosclerosis, hypertension and restenosis. Therefore, the inhibition of inflammatory factor and cytokine-induced VSMC proliferation and migration appears to be a promising therapeutic strategy for atherosclerosis, hypertension and restenosis. The regulatory role of AS-IV has also been reported in other cell types. Li *et al* showed that AS-IV regulated the cell proliferation of rat keratinocytes via mediating the Wnt signaling pathway (16). However, no previous study has reported the effect of AS-IV on VSMC proliferation. In the current study, AS-IV was demonstrated to have an inhibitory role in PDGF-BB-stimulated HDVSMC proliferation. Furthermore, as cell cycle-associated proteins are key regulators in cell proliferation, the expression levels were further investigated. The observations revealed that pretreatment with AS-IV significantly attenuated PDGF-BB-stimulated upregulation of the protein expression levels of cyclin D1, cyclin E, CDK2 and CDK4. Accordingly, these observations preliminarily indicated that AS-IV inhibits PDGF-BB-induced HDVSMC proliferation via regulating the expression of cell cycle-associated proteins.

Under normal conditions, VSMCs exhibit a differentiated phenotype; however, under stimulations, such as vascular injury or inflammatory responses, VSMC dedifferentiate into a proliferative phenotype (17,18). In addition, PDGF-BB has been reported to play a stimulatory role in the regulation of this phenotype switch (19,20). Accordingly, the effect of AS-IV on the PDGF-BB-stimulated phenotype switch of HDVSMCs was further investigated. The observations demonstrated that following administration of PDGF-BB, the expression levels of smooth muscle markers, including α-SMA, smoothelin and desmin, were significantly downregulated, indicating that HDVSMCs dedifferentiated into a proliferative phenotype. However, AS-IV effectively restored the expression levels, indicating that AS-IV inhibited the PDGF-BB-induced phenotype switch of HDVSMCs. These observations were consistent with the aforementioned results that AS-IV suppressed PDGF-BB-stimulated HDVSMC proliferation.

Abnormal migration of VSMCs also functions as a key promoter in neointima formation, which is closely associated with atherosclerotic lesions and restenosis following PCI (21,22). In addition, PDGF-BB has been reported to induce an increase in VSMC migration (23). Since AS-IV has been found to play a protective role in the cardiovascular system (2), AS-IV was hypothesized to exhibit a suppressive effect on the PDGF-BB-induced upregulation of VSMC migration. The results demonstrated that following PDGF-BB treatment, the migration of HDVSMCs was significantly upregulated, together with increased expression levels of MMP2 and MMP9, which is consistent with the results of previous studies (24,25). In addition, AS-IV markedly suppressed the PDGF-BB-stimulated upregulation of HDVSMC migration and attenuated the upregulation of MMP2. Therefore, the inhibitory effect of AS-IV on PDGF-BB-stimulated HDVSMC migration may be via the suppression of MMP2 upregulation.

The p38 MAPK signaling pathway has been demonstrated to be involved in the inflammatory response, which is a crucial pathogenic factor in cardiovascular disorders (26,27). In addition, the p38 MAPK signaling pathway participates in the regulation of VSMC proliferation by modulating the expression of cell cycle-associated proteins (28). Furthermore, this signaling pathway is associated with VSMC migration (29). In the present study, under the stimulation of PDGF-BB, this signaling pathway was shown to be activated, as demonstrated by the upregulation of phosphorylated p38 MAPK expression, which is consistent with the results of previous studies (19,30). However, pretreatment with AS-IV markedly inhibited PDGF-BB-induced p38 MAPK signaling activation. Accordingly, the suppressive role of AS-IV in PDGF-BB-stimulated HDVSMC proliferation and migration may be explained by the inhibitory effect on the activation of the p38 MAPK signaling pathway.

In conclusion, the current study demonstrated that AS-IV exhibits inhibitory effects on PDGF-BB-induced HDVSMC proliferation and migration. Molecular mechanism investigation revealed that the p38 MAPK signaling pathway is involved. Therefore, AS-IV may be useful for the prevention of neointima formation.

## Figures and Tables

**Figure 1:** AS-IV inhibited PDGF-BB-induced HDVSMC proliferation. MTT assays were performed to determine the rate of HDVSMC proliferation in each group. Control, HDVSMCs without any treatment; PDGF-BB, HDVSMCs treated with PDGF-BB; PDGF-BB + AS-IV, HDVSMCs treated with PDGF-BB and AS-IV; AS-IV, astragaloside IV; PDGF, platelet-derived growth factor; HDVSMC, human dermal vascular smooth muscle cell.

**Figure 2:** AS-IV suppressed PDGF-BB-induced upregulation of cell cycle-associated proteins in HDVSMCs. Western blot analysis was performed to determine the expression levels of cell cycle-associated proteins in each group. GAPDH was used as an internal reference. ^**^P<0.01. Control, HDVSMCs without any treatment; PDGF-BB, HDVSMCs treated with PDGF-BB; PDGF-BB + AS-IV, HDVSMCs treated with PDGF-BB and AS-IV; AS-IV, astragaloside IV; PDGF, platelet-derived growth factor; HDVSMC, human dermal vascular smooth muscle cell.

**Figure 3:** AS-IV suppressed the PDGF-BB-induced switch of HDVSMCs into a proliferative phenotype. Western blot analysis was performed to determine the protein expression levels of muscle cell markers in each group. GAPDH was used as an internal reference.^**^P<0.01. Control, HDVSMCs without any treatment; PDGF-BB, HDVSMCs treated with PDGF-BB; PDGF-BB + AS-IV, HDVSMCs treated with PDGF-BB and AS-IV; AS-IV, astragaloside IV; PDGF, platelet-derived growth factor; HDVSMC, human dermal vascular smooth muscle cell; α-SMA, α-smooth muscle actin.

**Figure 4:** AS-IV attenuated PDGF-BB-induced HDVSMC migration. Transwell assays were performed to determine the rate of HDVSMC migration in each group. ^**^P<0.01. Control, HDVSMCs without any treatment; PDGF-BB: HDVSMCs treated with PDGF-BB; PDGF-BB + AS-IV, HDVSMCs treated with PDGF-BB and AS-IV; AS-IV, astragaloside IV; PDGF, platelet-derived growth factor; HDVSMC, human dermal vascular smooth muscle cell.

**Figure 5:** AS-IV inhibited PDGF-BB-induced upregulation of MMP2 protein expression in HDVSMCs. Western blot analysis was performed to determine the protein expression of MMP2 and MMP9 in each group. GAPDH was used as an internal reference. ^**^P<0.01. Control, HDVSMCs without any treatment; PDGF-BB, HDVSMCs treated with PDGF-BB; PDGF-BB + AS-IV, HDVSMCs treated with PDGF-BB and AS-IV; AS-IV, astragaloside IV; PDGF, platelet-derived growth factor; HDVSMC, human dermal vascular smooth muscle cell; MMP, matrix metalloproteinase; ns, not significant.

**Figure 6:** AS-IV suppressed PDGF-BB-induced activation of the p38 MAPK signaling pathway in HDVSMCs. Western blot analysis was performed to determine the protein expression levels of phosphorylated p38 MAPK, as well as the total p38 MAPK expression level, in each group. GAPDH was used as an internal reference. ^**^P<0.01. Control, HDVSMCs without any treatment; PDGF-BB, HDVSMCs treated with PDGF-BB; PDGF-BB + AS-IV, HDVSMCs treated with PDGF-BB and AS-IV; AS-IV, astragaloside IV; PDGF, platelet-derived growth factor; HDVSMC, human dermal vascular smooth muscle cell; MAPK, mitogen activate protein kinase.
